# Influence of Nano-Cutting Fluid in New Cutting and Forming Processes on Heat Transfer Performance of Mechanical Engineering

This article has been retracted.

**DOI:** 10.1155/2022/5603355

**Published:** 2022-06-30

**Authors:** Wei Liu

**Affiliations:** Hebei Chemical & Pharmaceutical College, Shijiazhuang 050026, China

## Abstract

In order to strengthen the thermal conductivity of green cutting fluid and the influence of nano-cutting fluid from new cutting and forming processes on heat transfer performance of mechanical engineering, a research method was proposed based on the influence of nano-cutting fluid from new cutting and forming processes on heat transfer performance of mechanical engineering. The dispersion stability, thermal conductivity, and viscosity characteristics of the nanofluid were studied, and the effects of acidification treatment time, type and concentration of carbon tube particles, surfactants, and testing conditions on the above properties were analyzed. It was found that the filling rate of T321 was about 25% when CNTs were filled, and the optimal compounding ratio of the two surfactants, sodium dodecyl benzenesulfonic acid (SDBS) and Tween-80 (TW-80), for the preparation of stable dispersed nanofluids was 3 ∶ 7. The optimum ratio of compound active agent to carbon tube is 5 ∶ 1. When CNTs were acidified for about 9 h and dispersed in sufficient and stable condition, the thermal conductivity of the base liquid was increased by 110% by the composite, and the shape factor of CNTs had the most significant effect on the thermal conductivity. It was found that the composite nanofluids had higher thermal conductivity and lower viscosity than the nanofluids prepared by ordinary CNTs. This was due to the fact that surfaces of CNTs were chemically modified during the opening and internal filling process, so that the composite had better dispersion stability in the base fluid.

## 1. Introduction

Metal cutting is an important part of machinery manufacturing industry. It is estimated that metal cutting takes up about 30∼40% of the total mechanical processing [1], and the mechanical processing is mainly turning and grinding. In order to reduce cutting temperature, prolong tool life, and improve workpiece surface quality and dimensional accuracy, cutting fluid is widely used in metal cutting. In the metal cutting process, the main role of cutting fluid is lubrication and cooling, so as to prolong the tool life. According to the principle of metal cutting, the cooling and lubrication effect of cutting area is the main factor affecting the tool life. In the process of machining, the cooling and lubrication effect of the cutting area is poor, which not only increases the surface temperature of the cutting tool and aggravates tool wear but also reduces the machining accuracy [2]. Therefore, it is very important to reduce cutting force, speed up cooling, reduce cutting heat, reduce friction coefficient on friction surface, and use cutting fluid reasonably. Cutting fluid is one of the core components of metal cutting process system. It is widely used in high-precision turning, broaching, milling, and grinding. The wetting and lubrication characteristics of the “cutter-chip-workpiece” contact surface, as shown in Figure 1, are directly related to the cooling, lubrication, cleaning, and anticorrosion of the cutting process. The complex “solid-liquid-gas” interface physicochemical interactions across the millimeter-micron-nano-atomic/molecular scales are involved, and it is not easy to be detected and controlled in real time and has always been the difficulty of achieving high efficiency, high precision, and green in metal cutting. How to describe the wetting and lubrication characteristics of cutting fluid to “tool-workpiece-chip” in detail so as to reveal the mechanism of cutting fluid more effectively, so as to reduce the cutting force and friction and wear of the tool, and how to improve the environmental friendliness (green) and machining accuracy of cutting fluid is one of the urgent tasks in metal cutting industry.

## 2. Literature Review

Zahoor et al. prepared graphene nanocomposite films based on 1-octyl-3-methylimidazolimide liquid and graphene. The addition of graphene improves the bonding strength of the liquid and reduces the friction coefficient. Graphene nanoparticles act as nano ball bearings between interfaces. In the case of heavy load of graphene, nanoparticles are subjected to shear force, resulting in dislocation of their internal lattice and forming a lubricating system to reduce friction [3]. Khanna et al. prepared polytetrafluoroethylene/go nanocomposites that exhibit ultralow wear rates. Since the actual machined contact surface is uneven, and oxidized graphene fills the cracks and pits in the material, the repaired friction surface becomes relatively smooth and flat [4]. As and Diwakar pressed and burned graphene sheets into massive graphene by sintering method. When 3 N load was applied, the blocks almost had no wear marks, mainly because the graphene at the friction pad was subjected to external compression and densification with excellent lubrication performance. By adding graphene to liquid lubricants, the friction coefficient of lubrication is reduced and load carrying capacity is improved. Graphene forms a physical adsorption film because of its high surface potential energy or because positive and negative charges are attracted to each other during friction. In addition, oxidation chemical reaction occurs between nanoparticles and the surface of friction material, forming chemical protective film to achieve the friction reduction effect [5]. As and Diwakar studied the tribological properties of poly *α*-olefin lubricating oil blended with oleic acid-modified graphene and found that graphene could significantly improve the extrusion performance and bearing capacity and reduce the diameter of wear spot. It is conducive to the formation of physical adsorption film and self-healing film on the surface of friction pair to repair the wear surface [5].

Carbon nanotubes (CNTs) are made from single or multiple layers of graphite sheets that are curled around a surface at an angle [6]. The thermal conductivity of carbon nanotubes can reach 6000 W/(m·k), which is a very good thermal conductivity material. The cavity structure of carbon nanotubes can be filled with other materials under certain circumstances, thereby changing the thermal conductivity, electrical properties, magnetic properties, and behavior of carbon nanotubes [7]. A nano-cutting fluid was prepared by using CNT composites filled with lubricants as additives. On the one hand, the thermal conductivity of the cutting fluid could be further enhanced; on the other hand, lubricants in the composites could be released in the cutting area, which could play a better lubrication role. In this article, a typical high pressure lubricant additive (T321) was selected. Nanofluids prepared from mixtures of CNTs and T321 have been used as research materials to study the properties of nanofluids such as dispersion safety, thermal conductivity, and dynamic viscosity. The effects of acidification treatment, surfactant, component concentration, temperature, and other factors on the performance of nanofluids were analyzed to provide a theoretical basis for the practical application of this new nano-cutting fluid [8].

## 3. Research Methods

First, the complex of CNTs and T321 was prepared by the liquid phase wet chemical method, mainly in the following two steps [9]. (1) In the acidification treatment of CNTs, 20 g CNTs were added in a 1 L three-way flask with 800 mL of concentrated nitric acid, concentrated sulfuric acid, and hydrogen peroxide mixture (volume ratio 3 : 1 : 1, then 1 : 1 dilution). The mixture was stirred with magnetic force (500r/min) and condensed under water bath at 80°C for 3–12 h. After reflux, vacuum filtration was carried out. After drying at 80°C, the filter cake was ground into nanosized particles for 8 h, and acidified CNTs were obtained. (2) Preparation of complex: 7.5 g of T321 was dissolved in 300 mL of acetone and 10 g acidified CNTs were put in, and the mixture was put into a spherical flask for vacuumization (vacuum degree: −0.06 mpa). The mixture was ultrasonic under this condition for 6 h, and the temperature was 60°C. Finally, the filter cake is pumped and repeatedly cleaned with acetone to remove the unfilled T321. The filter cake was dried at 80°C and then ball milling for 8 h. CNT composites could be prepared [10]. There is unfilled T321 in the filtrate. After the acetone is dried, the unfilled T321 can be obtained and the mass can be measured, and the filling rate can be calculated by comparing it with the feed amount. The microstructure and written morphology of the samples were analyzed by TEM with a rated current of 200 kV. Thermogravimetric analysis was used to determine the temperature of carbon nanotube composites. The temperature was raised from 30°C to 600°C, and the heating was set at 20°C/min. The difference in absorption characteristics of carbon nanotubes before and after collection was detected by an infrared spectroscopy, and the samples were pressed with KBr. Secondly, nonionic surfactants AEO-5, OP-10, and TW-80 and anionic surfactants SDS-1, SDS-2, and SDBS were used as dispersion media to prepare nanoliquid solutions. Excluding other additives, the basic formula is surfactant (surfactant) + isocarbon. The specific method is to take a certain mass of active agent and dissolve it in water to prepare the base liquid of different concentrations, and then, take a certain mass of acidified CNTs or complex and add it to the corresponding base liquid. After ultrasonic treatment at 50°C for 1 h and mechanical stirring for 30 min, fully dispersed nanofluid with each volume of 100 mL is prepared [11].

After preparation, the nanofluid was left standing for 30 days, 1 mL of the upper liquid was taken every day, diluted twice, and put into a colorimetric dish to test the absorbance of the system at 500 nm wavelength. The stable value of absorbance is taken as the basis to judge the dispersion stability of the system.

Firstly, the absorbance of the nanofluid with the surfactant and carbon tube mass fraction of 0.1% was measured to judge the dispersion effect of different surfactants. The absorbance of the nanofluid with the ratio of nonionic and anionic surfactants (1 ∶ 9) to (9 ∶ 1) and the carbon tube mass fraction of 0.1% was determined to optimize the surfactant formulation. The absorbance of nanofluids with carbon tube mass fraction of 0.1% and complex active agent mass fraction of 0.02% ∼ 1.2% was measured to determine the appropriate concentration of complex active agent [12]. The above test temperature was 20°C, and CNTs were acidified for 6 h.

Secondly, the absorbance of nanofluid with 0.5% compound active agent and 0.02%–1.6% carbon tube (6 h) mass fraction was determined to investigate the influence of carbon tube concentration on the dispersion stability of nanofluid. The absorbance of nanofluid with compound surfactant mass fraction of 0.5% and carbon tube mass fraction of 0.1% was measured. In this case, the acidification treatment time of CNTs was 3 h, 6 h, 9 h, and 12 h, respectively, to investigate the influence of carbon tube aspect ratio on dispersion stability. The above tests were carried out at 20°C.

Finally, TC3010L thermal conductivity meter (transient hot wire method) was used to measure the thermal conductivity of the above groups of samples, and the samples to be tested were used to wash the sample tank before each test. Each test requires about 30 mL of the sample, and the instrument automatically determines the thermal conductivity value after the completion of sample injection. The dynamic viscosity of nanofluids was measured by ndJ-5S viscosimeter with rotor no. 1 at 12r/min. Firstly, the effects of the mass fraction of carbon tube (0.02% ∼ 0.6%), the mass fraction of compound surfactant (0.02% ∼ 1.2%), and the acidification treatment time of CNTs (3 h, 6 h, 9 h, and 12 h) on the thermal conductivity and dynamic viscosity were tested at 20°C. The thermal conductivity and viscosity of the nanofluids were tested when the temperature was 20 ∼ 80°C, the mass fraction of the compound active agent was 0.5%, and the mass fraction of carbon tube was 0.1%.

## 4. Result Analysis

### 4.1. Characterization of CNTs Complex

Figure 2 shows the infrared spectra of CNTs, acidified CNTs, T321, and complex. As can be seen from Figure 2(a), new absorption peaks of CNTs appeared near 3632 cm^−1^ and 1722 cm^−1^ wavelengths after acidification, which should be attributed to hydroxyl and carboxyl groups, etc., indicating that oxygen-containing groups were bonded by acidified CNTs. This has a good effect on improving the dispersion stability of CNTs in the base liquid. In addition, the peak value near 1543 cm^−1^ should be attributed to the planar absorption peak of the carbon ring structure, which proves that CNTs retain their own tubular structure, and this is a prerequisite for filling the tube with T321 [13]. As shown in Figure 2(b), no new characteristic peak was detected in the infrared spectrum of the CNTs complex, and the characteristic peak was the partial superposition of the characteristic peak of acidified CNTs and T321, proving that the physical bond between the two had mainly occurred during the filling of CNTs by T321, instead of a chemical reaction.

The state of T321 in CNT tube can be directly determined by TEM observation of the microstructure of carbon tube. There was a shadow area on the end face of acidified CNTs because after CNTs were truncated by acidification, the carbon tube end face was bonded with functional groups such as carboxyl group and hydroxyl group, which increased the carbon content at the end face. Several sections of the carbon tube are obviously wetted by T321, which intuitively proves the existence of T321 in the tube [14].

In addition, thermal analyses of CNTs, acidified CNTs, and CNT composites were performed. It can be seen from Figure 2(a) that the thermogravimetric curves of carbon nanotubes and acidified carbon nanotubes are similar, and the thermogravimetric processes are also similar. However, the thermogravimetric curves of carbon nanotube composites have obvious weight loss processes at lower temperatures, which should be the result of T321 escaping from the complex, and it also proves the presence of T321 inside the CNT tube. The filling rate of T321 in CNTs can be calculated according to equation (*η*):

(1) $$\begin{array}{c} \eta =\frac{H_{f}}{H_{p}}\times 100\%. \end{array}$$

Here, *H*_*f*_ is the latent heat of phase transition of T321 filled in CNTs, J/g, and *H*_*p*_ is the latent heat of T321, J/g.

The DSC curve of the composite shown in Figure 3 shows that the latent heat of phase change of T321 is 31.58 J/g, while that of T321 under the same conditions is 123.24 J/g. Therefore, the filling rate of T321 in CNTs can be calculated as 25.6%. In addition, by drying the acetone in the filtrate extracted from the compound and weighing the weight of the remaining T321, the filling rate of carbon tube can be calculated to be about 25%, which is basically consistent with the analysis result of DSC [15].

### 4.2. Dispersion Stability of Nanofluids

#### 4.2.1. Influence of Surfactant

Nanofluids of CNT composite prepared by six surfactants (standing for 1 day) were utilized. Fluid no. 1 was prepared with untreated CNTs and the active agent was TW-80. No. 2–7 were prepared from CNT complex with active agents of MOA-5, OP-10, TW-80, SDS-1, SDS-2, and SDBS. The dispersion of tw-80 nanofluids prepared from untreated CNTs showed significant agglomeration while there was no agglomeration in nanofluids of CNTs composite [16]. This is because after the carbon tube is acidified, its length-diameter ratio becomes smaller, which makes the contact area between the carbon tube become smaller and it is not easy to entangle. In addition, after acidification, the carboxyl and hydroxyl groups bonded at the end of carbon tubes reduce the van der Waals force between carbon tubes, and make the surfactant more easily bonded with carbon tubes, and enhance the steric hindrance between carbon tubes. Carbon tubes mostly exist in the form of single root, which also proves that the nanofluid of CNTs composite has good dispersion under the action of surfactants.

Among the three nonionic surfactants, MOA-5 has the best dispersibility, TW-80 has the best dispersibility, followed by OP-10. The nonionic active agent disperses the carbon tube only through the steric hindrance of the polar chain. The longer and more complex the molecular chain, the better the dispersion effect. Tw-80 has the longest chain and three segments of hydrophilic polyoxyethylene on each molecule. MOA-5 and OP-10 have short molecular chains and low hydrophilicity of polyoxyethylene, so TW-80 has the best dispersion effect. There is a benzene ring in the molecular structure of OP-10, which may be in contact with carbon tubes, so its dispersibility is better than that of MOA-5 [15]. In summary, TW-80 is the best choice among the three nonionic active agents. In addition, sdS-2 and SDBS of the three anionic active agents have good dispersion effect on carbon tube, which is due to the obvious Coulomb attraction between anionic active agent and the opposite charge on the surface of carbon tubes. The molecular structure of SDS-1 and SDS-2 are almost identical, but the dispersion of SDS-1 is poor, which may be caused by the larger critical micelle concentration (CMC) of SDS-1.

Some studies have shown that the combination of nonionic and anionic surfactants can achieve better dispersion effect. Therefore, SDS-2 and SDBS were used to compound TW-80 in this article, and it is known that the optimal dispersion effect can be achieved when the ratio of SDBS to TW-80 is 3 : 7 [17]. This is because, compared with SDS-2, the benzene ring structure of SDBS has a stronger adsorption capacity for carbon tubes, and there is a synergistic effect between SDBS and TW-80, thus improving the dispersion effect.

Figure 4 shows the influence of the mass concentration of the preferred compound active agent on the absorbance of the system (the mass fraction of carbon tube is 0.1% at this time). It can be seen that when the concentration of active agent is in a lower range, the absorbance of the system continues to increase. When the mass fraction of active agent increases to about 0.5%, the carbon tube is completely dispersed and the system is in a state of “saturation.” The absorbance of the system was little changed by increasing the concentration of active agents. Therefore, it can be judged that the best mass ratio of compound surfactant to carbon tube is 5 : 1.

#### 4.2.2. Influence of Carbon Tube Mass Fraction and Acidizing Treatment Time

Figures 5(a) and 5(b) show the influence of carbon tube concentration on absorbance when the mass fraction of compound active agent is 0.5%. It can be seen that when the concentration of carbon tubes is small, the absorbance increases gradually with the increase of pressure, and the relationship is linear. However, the absorbance did not increase much when the carbon tube concentration reached the “saturated” concentration, which was due to the uniformity of some poorly dispersed carbon tubes [18]. Furthermore, it was found that under the same conditions, the stability of carbon nanotube composites was better than that of acidified carbon nanotubes, which may be due to the fact that the exposed T321 molecular groups of carbon tubes were mixed with surfactants to improve dispersion.

The acidification treatment can cut the carbon nanotubes into shorter tubes, and the longer the acidification time, the smaller the ratio, which also affects the function of the nanofluid.  Figure 5(b) shows the effect of acidification time on the absorbance of the system when the main component of active compound is 0.5% and the main component of carbon tube is 0.1%. It can be seen that the absorbance increases with the increase of treatment time. This is because the agglomeration and entanglement between carbon tubes weaken and the number of end faces increases with the decrease of the aspect ratio. The more oxygen-containing groups are bonded, the more obvious the dispersion effect of surfactant on carbon tubes is. However, if the aspect ratio is too small, the carbon tube is too short to fill and store lubricant. According to the corresponding relationship between the acidification treatment time of carbon tubes and the ratio of length to diameter, combined with the results in Figure 5(b), it is preliminarily judged that the acidification treatment time of carbon tubes used in this article is about 9 h.

### 4.3. Thermal Conductivity of Nanofluids

#### 4.3.1. Influence of Carbon Tube and Surfactant Mass Fraction

The thermal conductivity of carbon nanotubes is higher than that of other nanoparticles, which can improve the thermal conductivity of the working fluid medium. Therefore, carbon nanotubes have great potential for improving heat transfer in liquids. When the volume of the working mixture is 0.5%, the thermal conductivity increases with the concentration. Compared with the thermal conductivity of the base liquid when the volume fraction of the composite active agent is zero, the composite material can increase the thermal conductivity of the base liquid by 110%. When the mass fraction of the carbon tube is 0.1%, the influence of the concentration of the compound active agent on the thermal conductivity is obvious when the concentration of active agent is low, but the effect of increasing the concentration of active agent on the thermal conductivity is limited. This is because the more carbon per unit volume is dispersed in the nanofluid, the stronger the Brownian motion, the higher the thermal conductivity of the object, and the more carbon remaining. Therefore, the thermal conductivity of nanofluids can be improved only by stabilizing carbon tubes dispersed in the base liquid.

#### 4.3.2. Influence of Carbon Tube Acidification Treatment Time and Test Temperature

When the mass fraction of carbon tube is 0.5% and the mass fraction of compound active agent is 0.1%, the thermal conductivity reaches the maximum when the treatment time is 9 h, and too long acidification time is not beneficial to the improvement of thermal conductivity. The complete existence of carbon tube structure after acidification and filling treatment has been proved by IR and TEM analysis. After dispersing into the base liquid, the smaller the proportion of carbon tubes, the more dispersed in the base liquid, the more effectively the thermal conductivity of the system can be improved. But if the sample is too short, it will affect the thermal conduction channel of the carbon tube and reduce the thermal conductivity of the system. Therefore, the proper acidification treatment time can make the nanofluids have good dispersion stability and thermal conductivity. The optimal acidizing time of carbon tube is 9 h.

When the mass fraction of carbon tube is 0.5% and the mass fraction of active agent is 0.1%, the effect of temperature on thermal conductivity is tested. When the temperature is lower than 60°C, the thermal conductivity can be improved by increasing the temperature due to the strong molecular motion. When the temperature is above 60°C, the thermal conductivity is not significantly improved. In addition, nanofluids with CNT composite showed better thermal conductivity due to the better dispersion of the composite in the base fluid, which is conducive to heat conduction [19]. There are many theoretical explanations for the mechanism of nanoparticles improving the thermal conductivity of nanofluids, such as Brownian motion of particles, suspension properties, and nanoliquid film. People have also proposed many thermal conductivity calculation formulas, such as H-C model, as shown in the following equation:

(2) $$\begin{array}{c} \frac{k_{\text{eff}}}{k_{f}}=\frac{k_{p}+\left(n-1\right)k_{f}-\left(n-1\right)f\left(k_{f}-k_{p}\right)}{k_{p}+\left(n-1\right)k_{f}+f\left(k_{f}-k_{p}\right)}, \end{array}$$

where *k*_eff_ is the thermal conductivity of the nanofluid; *k*_*f*_ is the thermal conductivity of the base liquid; *k*_*p*_ is the thermal conductivity of nanoparticles; f is particle volume fraction; and *n* is the empirical shape factor (spherical shape *n* = 3, cylindrical shape *n* = 6). In the formula, both *k*_*f*_ and *k*_*p*_ are known values. The density of carbon tubes in this article is about 1.8 g/cm3, based on which the value of *f* can be calculated.

When *n* and kp of CNT complex are set at different values, the theoretical values of thermal conductivity of nanofluids under different volume fractions are calculated by the H-C model. When the shape factor *n* = 5, the theoretical values calculated by H-C model are in good agreement with experimental data. Therefore, the theoretical calculation formula of thermal conductivity of nanofluids is shown as follows:

(3) $$\begin{array}{c} \frac{k_{\text{eff}}}{k_{f}}=\frac{\left(1+4f\right)k_{p}+4\left(1-f\right)k_{f}}{\left(1-f\right)k_{p}+\left(4+f\right)k_{f}}. \end{array}$$

By calculating the sphericity of the carbon tube, the shape factor *n* is 25, but the value of *n* decreases after the carbon tube is dispersed into the base solution. In H-C formula, *n* mainly affects the value *k*_eff_, and *k*_*p*_ has little influence. Therefore, it is the key to improve the thermal conductivity of nanofluids by further improving the dispersion of complex in the base liquid and increasing the value of its shape factor in the nanofluids.

## 5. Conclusion

1. The acidified carbon nanotubes are excised, but the tubular structure is preserved, and the final surface is modified. The effective acidification time of CNTs was 9 h. T321 was successfully incorporated into acidic carbon nanotubes and was developed with a fill rate of approximately 25%.
2. The optimum ratio of SDBS and TW-80 for the preparation of stably dispersed nanofluids is 3 ∶ 7. The optimum ratio of compound active agent to carbon tube is 5 ∶ 1. The CNT complex increased the thermal conductivity of the base liquid by 110% under stable and fully dispersed conditions.
3. Nanofluid formulations are non-Newtonian liquids. The viscosity of the nanofluidic formulation was lowest when the volume of the surfactant complex was about 0.5%. Compared with acidified carbon nanotubes, nanofluids prepared from carbon nanotube composites have higher thermal conductivity and lower viscosity. This is due to the chemical modification of the surface during the opening and interior filling of CNTs, which provides better dispersion stability of the complexes in the base fluid.

## Figures and Tables

**Figure 1:** Mechanical manufacturing flowchart.

**Figure 2:** (a) CNTs. (b) Complex.

**Figure 3:** TG and DSC thermogravimetric analysis of CNTs, acidified CNTs, and CNTs complex.

**Figure 4:** Influence of mass fraction of complex surfactant on absorbance of the system.

**Figure 5:** (a) Influence of carbon tube concentration. (b) Acidizing time.

## Data Availability

The data used to support the findings of this study are available from the corresponding author upon request.
